# Assessment of Effective Network Connectivity among MEG None Contaminated Epileptic Transitory Events

**DOI:** 10.1155/2021/6406362

**Published:** 2021-12-28

**Authors:** Abir Hadriche, Ichrak Behy, Amal Necibi, Abdennaceur Kachouri, Chokri Ben Amar, Nawel Jmail

**Affiliations:** ^1^REGIM Lab, ENIS, Sfax University, Tunisia; ^2^Digital Research Center of Sfax, Tunisia; ^3^MIRACL Lab, Sfax University, Tunisia; ^4^LETI Lab, ENIS, Sfax University, Tunisia

## Abstract

Characterizing epileptogenic zones EZ (sources responsible of excessive discharges) would assist a neurologist during epilepsy diagnosis. Locating efficiently these abnormal sources among magnetoencephalography (MEG) biomarker is obtained by several inverse problem techniques. These techniques present different assumptions and particular epileptic network connectivity. Here, we proposed to evaluate performances of distributed inverse problem in defining EZ. First, we applied an advanced technique based on Singular Value Decomposition (SVD) to recover only pure transitory activities (interictal epileptiform discharges). We evaluated our technique's robustness in separation between transitory and ripples versus frequency range, transitory shapes, and signal to noise ratio on simulated data (depicting both epileptic biomarkers and respecting time series and spectral properties of realistic data). We validated our technique on MEG signal using detector precision on 5 patients. Then, we applied four methods of inverse problem to define cortical areas and neural generators of excessive discharges. We computed network connectivity of each technique. Then, we confronted obtained noninvasive networks to intracerebral EEG transitory network connectivity using nodes in common, connection strength, distance metrics between concordant nodes of MEG and IEEG, and average propagation delay. Coherent Maximum Entropy on the Mean (cMEM) proved a high matching between MEG network connectivity and IEEG based on distance between active sources, followed by Exact low-resolution brain electromagnetic tomography (eLORETA), Dynamical Statistical Parametric Mapping (dSPM), and Minimum norm estimation (MNE). Clinical performance was interesting for entire methods providing in an average of 73.5% of active sources detected in depth and seen in MEG, and vice versa, about 77.15% of active sources were detected from MEG and seen in IEEG. Investigated problem techniques succeed at least in finding one part of seizure onset zone. dSPM and eLORETA depict the highest connection strength among all techniques. Propagation delay varies in this range [18, 25]ms, knowing that eLORETA ensures the lowest propagation delay (18 ms) and the closet one to IEEG propagation delay.

## 1. Introduction

Diagnosis of neurologic disease is oriented now days, into exploring noninvasive modalities as electroencephalography (EEG) and magnetoencephalography (MEG) techniques [1]. In fact, EEG and MEG recordings allow high time and space precision in featuring brain function and dysfunction especially in epilepsy diagnosis.

Major feature that may predispose advantages of MEG on EEG is the fact that MEG requires less detail about cortical tissue in order to define sources and epileptic seizure [2]. Hence, and despite its cost, neurologist and biomedical researchers are using MEG as a complementary way to diagnosis epilepsy. Especially, for pharmacoresistant one to manage placement of intracranial EEG (as intracerebral EEG), to overcome and limit surgical intervention [3]. Pharmacoresistant epilepsy requires a highly space precision to define epileptogenic zones (EZ) [4, 5] which would be restricted through a surgical intervention. Alternatively, several cerebral regions could be implicated, either as propagation areas or as generator of epileptic discharges [6]. Therefore, neurologists rely on network connectivity of MEG hallmark signals (high frequency oscillations (HFO), gamma oscillations [7], ripples, and transitory activities [4]) in order to detect accurate EZ [8]. However, these activities (transitory and oscillatory) are mutually contaminated due to overlap in time frequency plane [9]. Defining efficiently, their spatiotemporal features is a fragile task, especially, using a classical band pass filter which generates spurious oscillations and false ripples [9]. This would affect obviously accurate definition of cortical malformation [10] and build-up of a seizure. In a previous work, we proposed and evaluated performances of several filtering techniques in separation between transient and oscillatory activities (matching pursuit (MP), finite impulse response filter (FIR), and stationary wavelet transform (SWT)) [11, 12], to recognize build-up seizure and EZ [5, 13].

Here, we suggest to evaluate robustness of an advanced methods based on Singular Value Decomposition (SVD) technique [14] in recovering pure epileptic transitory activities none contaminated by gamma oscillations among MEG signals. An advanced method of rebuilding pure interictal epileptiform discharges is based on a decomposition algorithm of transitory events generating suited basis. We projected our studied signal on these transitory bases, followed by a thresholding step (applied on resulting transitory component). Finally, a recovery phase is applied that reassembles only accurate selected components (transitory one) [15].

In this study, we simulated a signal with five different time transitory occurrences, depicting intermingled transient and ripple events for different frequency and signal to noise ratio. Our simulated data present both epileptic biomarkers (separated, overlapped, and fully overlapped) in respect with morphological and spectral features of realistic data. These simulated data will be an efficient solution to evaluate the separation between epileptic biomarkers and recognizing pure cortical generators.

We calculated reconstruction's goodness of fit GOF on behalf of the frequency range of ripples, transitory time occurrence, and SNR. We evaluated robustness of our advanced technique, through recognition and automatic detection of pure interictal epileptiform discharges using topography maps and precision measures among MEG signals. After validating our proposed separating technique's robustness in detecting and recovering pure epileptic transitory events, we proceeded in defining their network connectivity and confronting with IEEG networks.

The second aspect is about locating actual generators of pure interictal epileptiform discharges with source localization methods. Reconstructed temporal dynamics of cerebral regions of interest ROI (epileptic generators) is an efficient way to inspect dynamics of epileptic network activations. Thus, measuring connectivity using correlation, coherence, and Directed Transfer Function (DTF) would estimate interactions between different epileptic cortical regions [5]. In fact, MEG source connectivity is extensively studied to delineate functional brain networks at cortical level and epileptic networks (locate EZ by investigating neural networks of excessive discharges). We proceed firstly, with a source localization step by resolving forward and inverse problem. Several methods of inverse problem are proposed in the literature; each has its own advantages and disadvantages that suit a specific situation and case of study. Indeed, there are several solutions such as linear, distributed, instantaneous, and discrete solutions, which are able to locate active sources. Here, we suggested studying and evaluating four distributed inverse problem methods: MNE (Minimum norm estimation), dSPM (Dynamical Statistical Parametric Mapping), eLORETA (Exact low-resolution brain electromagnetic tomography), and cMEM (Coherent Maximum Entropy on the Mean) to distinguish neural networks involved in genesis of pure interictal epileptiform discharges. MNE and eLORETA proved an excellent accuracy in locating deep sources. dSPM presented good timing and spatial extent of language processes in epilepsy [16–18]. cMEM demonstrated a high precision in spatially spread of epileptic sources [19].

Finally, MEG epileptic networks are confronted to intracerbral networks by nodes in common, connection strength, distance of common nodes, recognition of seizure onset zone SOZ, and average propagation delay.

Three keys component are investigated in our study: capacity of recognition of pure transitory hallmark, evaluation of 4 inverse problem methods using network connectivity, and confrontation of scalp effective connectivity to intracerebral one. Three substudies are presented where we describe in the first substudy the automatic detector of pure transitory activities (pure neural epileptic transitory generator). In the second substudy, we applied 4 inverse problem techniques to compute network connectivity of MEG transitory events using cross-correlation measures. In the last part, we investigated inverse problem performances by confronting MEG network connectivity to invasive network connectivity. Our obtained results could be considered a prognosis to assist a neurologist during epilepsy diagnosis to recognize EZ.

## 2. Materials and Methods

### 2.1. Materials

#### 2.1.1. Simulation

We simulated a dataset inspired from real preprocessed MEG signals, validated by an experienced clinical neurophysiologist, with a sampling frequency equal to 1024 Hz. We produced patterns with a mixture between transitory and gamma oscillatory activities (both epileptic biomarkers), intermingled with a noncortical brain artefacts (ocular blink). Transitory activities are generated as a sum of two gamma functions, applying the gampdf (*x*, *a*, *b*) function in Matlab. Time variable in samples was adjusted as (*a*, *b*) to (9.8, 3.9) in channel 1, (7.8, 2) in channel 2, (11.7, 3.9) in channel 3, (11.7, 2) in channel 4, and (12.7, 2) in channel 5. Transitory amplitudes were equal to 10, with a uniform distribution of fluctuation (from 10% to 25%). Oscillations were procured as oscillatory pulses obtained by the gausspuls (*t*, fc, bw) function of Matlab; with *t* time, fc frequency of oscillations which is set to 45, 55 65, 75, and 85 Hz; bw fractional bandwidth equal to 0.15; and amplitude fluctuations of 25% in channel 3 and 15% in channel 4. On the other hand, we imposed a translation of ripple window across transitory window with equal steps. Hence, our simulation depicts transitory and ripples separated in time, overlapped, and fully overlapped [9]. We added a noise with a physiologically plausible 1/*f* spectrum, from a neural mass model [4]. SNR was calculated as 10 × log 10 (signal energy/noise energy); then, we varied SNR in this range [-5, 15, 20] dB. For each SNR value, we generated 100 realizations. We simulated five channels where we varied transitory time occurrences within equal steps across ripple time window (between 200 and 250 ms).

Each channel presents a mixture of transitory and ripples for a frequency range of [45, 55, 65, 75, 85] Hz. SNR values, transitory time occurrence, and frequency ranges affect directly the performances of reconstruction and automatic detection of pure transitory events. To address this issue, we evaluated the rate of pure epileptic transitory activities rebuilding in terms of SNR, transitory time occurrence, and frequency range. In total, by changing these parameters, we studied 7500 realizations (3∗SNR∗5 transitory time occurrence∗5 frequency∗100 realizations). In these simulated data, we produced signals respecting the same morphological, time series, and spectral proprieties as MEG signal, with 5 channels and 7500 trials of 300 ms in order to study robustness of our proposed advanced technique in defining pure epileptic transitory generators.

#### 2.1.2. Real Signal

Real explored signals were both MEG and IEEG for five pharmacoresistant subjects. Acquisition and preprocessing steps were applied in Clinical Neurophysiology Department of La Timone hospital in Marseille, France.

Five pharmacoresistant patients are selected by an expert neurologist (M.G.) depicting stable and frequent epileptic transitory activities (interictal epileptiform discharges). MEG signal was recorded on a 151-gradiometer system (CTF Systems Inc., Port Coquitlam, Canada), with eyes closed, no activation procedure nor movement. Sampling frequency was set to 1025 Hz, and 20 epochs of 5 s were recorded. Abundant transitory activities were registered that predispose studying pure transitory activities as a biomarker for epilepsy diagnosis as in [5]. Intracerebral EEG signals were gathered as Talairach stereoscopic method [20], sampled at 512 Hz. Seven to 16 multicontact depth electrodes (Alcis, Besancon, France) were implemented. Each electrode has 0.8 mm of diameter and 10 to 15 contacts of 2 mm long. Depth electrodes provide in total 70 to 128 measures. Clinical, neurophysiological, and anatomical features of each patient as in [5] were taken into consideration to designate cerebral marks.

An Optima CT 660 system of the General Electric Healthcare was used for the cerebral CT images, with 120 kV, 230-270 FOV, 512 × 512 matrix, and 0.6 mm slice thickness, without injection of contrast agents. Each CT scan was reconstructed using the standard (H30) reconstruction kernel to limit the level of streaks or flaring. For the MRI examinations, a 1.5 T system (Siemens, Erlangen, Germany) during the weeks before SEEG implantation was performed. Used MRI protocol included at least T1-weighted gradient-echo, T2-weighted turbo spin-echo, FLAIR images in at least two anatomic planes, and a 3D-gradient echo T1 sequence of 4 min, 16 seconds after gadolinium based contrast agents (GBCA) injection.

Promptly, a postoperative computed tomography scan and MRI were performed during the removal of depth electrode to double check accurate coordinate.

Interpretation and time series analysis of IEEG recording are achieved using bipolar montage. Patients signed informed consent, and the Institutional Review board (IRB00003888) of INSERM (IORG0003254, FWA00005831) approved the study. In Table 1, we gathered the patient's clinical background.

### 2.2. Methods

All simulated signals and signal processing were applied using the MATLAB (MathWorks, Inc.) software, Brainstorm, EEGlab [21], Fieldtrip toolbox, and LORETA software (free academic) [22].

#### 2.2.1. Detection of Transitory Shapes

To detect transitory activities among simulated and MEG signal, we proceeded as in [21]. We applied, for each channel separately (since transitory shape can change from a captor to another), a high and a low thresholding step on amplitude distribution *Q*_*p*_ of 0.5, 0.75, and 0.25 percentile, as explained in

(1) $$\begin{array}{c} {\text{thr}}_{h}=Q_{0.5}+d\left(Q_{0.75}-Q_{0.25}\right), \end{array}$$

(2) $$\begin{array}{c} {\text{thr}}_{l}=Q_{0.5}-d\left(Q_{0.75}-Q_{0.25}\right). \end{array}$$

We imposed a 10 ms distance between two consecutive peaks (inspired from trigging MEG epileptic transitory). Hence, we obtained local peaks of transitory among simulated and real data. We created transitory epochs around peaks with respect to distance constraints between two consecutive activities (10 ms).

#### 2.2.2. SVD

After automatic detection of transitory, we segmented our database (simulated and MEG signal) in events lasting 200 ms around detected peaks. Then, we performed SVD on these epochs and for each channel consecutively [14]. SVD is a preprocessing technique that creates a new signal through a specific number of components [23] (generators of transitory and oscillatory shapes). We covered thresholding steps to select only transitory components from oscillatory ones. SVD of a given signal **X** is **σ** that verifies

(3) $$\begin{array}{c} X*V=\sigma U,\\ X*U=\sigma V, \end{array}$$

where *X* is a matrix with (*m*, *n*) dimension, *U* is *n* left singular vector, and *V* is m right singular vector. SVD of *X* is a reduction of *X* to a bidiagonal matrix obtained through a product between 2 orthogonal columns *U*, *V*. ∑ is a diagonal matrix with a nonnegative value as defined in

(4) $$\begin{array}{c} X=U\;\Sigma \text{ V}. \end{array}$$

Hence, we created a new basis by exploring only the first three sum product of time *U*(*t*) and space *V*(*s*) components as in Equation (5) (first three components have a transitory shape that disappears from the fourth component and transforms into oscillatory events).

(5) $$\begin{array}{c} T\left(t\right)=\overset{3}{\underset{1}{\sum }}\underset{i}{\sum }u_{i}v_{i}. \end{array}$$

The last step of transitory recovering is projecting our original signal (simulated and MEG signal) on the new obtained suited transitory basis [5].

#### 2.2.3. GOF of Simulated Data

Goodness of fit (GOF) is a measure that reflects our advanced filtering technique robustness in reconstructing of pure transitory among original signal composed of a mixture of oscillations (ripples, HFO) and transitory [11, 24] events. GOF is a ratio between pure transitory activities energy per original signal energy as defined in Equation (6).

(6) $$\begin{array}{c} \text{GOF}=\frac{\sum {\left(x\left(t\right)-\hat{x\left(t\right)}\right)}^{2}}{\sum x{\left(t\right)}^{2}}, \end{array}$$

where *x*(*t*) is the original signal and $\hat{x\left(t\right)}$ is the recovered pure transitory activity.

We computed GOF for 7500 realizations in order to evaluate our advanced filtering technique efficiency in separation between ripples and transitory for different SNR, shapes, and frequency range.

For MEG signal, we added another preprocessing step before applying our advanced filtering technique, which is classification of epileptic transitory events based on its morphology and guided by an expert neurologist.

#### 2.2.4. Clustering MEG Transitory Activities

Epileptic transitory events were selected from first run of MEG signal by an expert neurologist (M.G.). Almost 50 events per patient were detected; however, these epochs did vary in shape from one channel to another as in [11]. Hence, we applied a clustering step to classify these transitory events sharing the same spatiotemporal shape (same active generators). A temporal translation was applied to align transitory peaks; then, the *k*-means algorithm was used for clustering [24]. An expert neurologist imposed 2 clusters [25]. We proceeded in the same way for the 5 studied patients as in [11].

#### 2.2.5. Precision of Pure Transitory Automatic Detector

As in [5, 11], an expert neurologist made a visual marking of epileptic transitory activities on MEG signal. Then, we performed automatic detection by our advanced technique [25] on local peaks (Section 2.2.1). Finally, we calculated precision *P* (see equation (7) to evaluate automated detector performances).

(7) $$\begin{array}{c} P=\frac{\text{TP}}{\text{TP}+\text{FP}}, \end{array}$$

where TP is true positive, FP is false positive, and *P* is precision measure of a deviation between true and false values [26]. To push ahead effectiveness of automatic epileptic transitory recognition and detection, a second precession *P* [27] was calculated on behalf a second guided human detection as in [13].

#### 2.2.6. Topography of Recovered MEG Transitory Events

To evaluate the capability of pure epileptic MEG transitory reconstruction, we averaged all selected transitory activities that belong to each cluster. Then, we compared topography of original signal versus detectable pure transitory. Topography maps were calculated on transitory event peaks. In fact, topography maps illustrate two-dimensional representations of multichannel on a scalp. Dipolar topography implies a cerebral activity. However, a random activity could be a result of noisy or induced noncortical activity depicting a random phenomenon [28].

#### 2.2.7. Source Localization of MEG Signal

*(1) Forward Problem*. Forward problem is a way to model the head, obtained through analytical or numerical methods as finite element method (FEM), boundary element method (BEM), and finite difference method (FDM). As our skull thickness is not homogeneous across the head, MRI is required to describe local conductivity properties. We resolved forward problem as in [5], shaping a multiple-sphere head model per subject. We used BrainVisa software, for segmentation and meshing of cortex and scalp surfaces. Finally, we adopted Brain storm toolbox on Matlab to register MRI and sensors of each studied subject [29].

*(2) Inverse Problem*. In order to understand cerebral function and dysfunction, we should define accurate sources that generate scalp measurement (MEG in our case) [30]. For epilepsy, we identify responsible regions of excessive discharges and build-up of a seizure (damaged cerebral tissue), by solving the inverse problem of localization sources. Since an inverse problem is a badly posed problem (different sources may generate identical potential field), there is no single solution. Hence, to reconstruct an efficient solution, we have to test and apply different assumptions (neurophysiological, biophysical, and anatomical) and regularization methods too. Dipolar source localization was explored as a solution, but assumption about the number of used dipole encourages researchers toward distributed techniques. These methods mainly concern a configuration of 3D current source solution grid with fixed positions. Moreover, distributed methods require only regularization parameters to limit noise effect and balance obtained source configuration. We choose to evaluate distributed inverse techniques since dipolar solution is penalized by the null hypothesis of source number. Moreover, it has been proved that MNE, dSPM, eLORETA, and cMEM are quite efficient in studying epilepsy and defining epileptogenic zones [31]. Next, we will describe briefly four distributed inverse problem methods (MNE, dSPM, eLORETA, and cMEM).

Minimum norm estimation (MNE) is proposed by [32]; it provides a unique solution of 3D current configuration which matches studied signal within a minimum intensity (smallest L2-norm). This assumption drowns deeper sources since MNE emphasizes superficial sources. The MNE formula is depicted in Expression 8.

(8) $$\begin{array}{c} S_{\text{MNE}=\;}G^{T}{\left({GG}^{T}+\lambda C\right)}^{-1}\;G, \end{array}$$

*C* is the noise covariance matrix, and *λ* displays the regularization parameter.

It is to remind that dSPM, eLORETA, and cMEM could be considered as weighted solution of MNE (their formula is based on MNE sources (*S*_MNE_)).

Dynamical Statistical Parametric Mapping (dSPM) is proposed by Dale et al. as another solution of the inverse problem. Inspired from MNE, Dale et al. suggest a normalization based on a minimum norm estimate of the noise (obtained from MNE noise covariance matrix) of each source [33, 34]. dSPM is considered a least-squares or weighted minimum norm solution, presented as

(9) $$\begin{array}{c} S_{\text{dSPM}}=W_{\text{dSPM}}S_{\text{MNE}},\\ W_{\text{dSPM}}^{2}=\mathrm{diag}\left(S_{\text{MNE}}\;CS_{\text{MNE}}^{T}\right). \end{array}$$

Exact low-resolution brain electromagnetic tomography (eLORETA) is proposed by Pascual-Marqui who introduced eLORETA as a zero error localization inverse problem solution [35]. The eLORETA method is a standard type of MNE with particular weights that use high space correlation between active neurons. eLORETA is efficient in the presence of structured noise and in finding superficial and deep sources too, considered an improvement over proposed tomographies LORETA and sLORETA.

Coherent Maximum Entropy on the Mean (cMEM) is demonstrated to be capable of finding hidden sources within a spatial extent. cMEM is a standard MEM with a stable location of clustering source in time domain, obtained by an optimal single patch of cortex as a spatial front. MEM is based on a probabilistic method approximating current source intensities from studied data. Grova et al. and Chowdhury et al. have extensively studied cMEM behaviour in presence of realistic simulations of EEG and MEG data; they assessed cMEM sensitivity to spatial generators extent. cMEM has shown good precision and robustness in reconstructing MEG sources of different sizes and depth [36, 37].

*(3) Evaluation and Comparison of Inverse Solutions*. After head modelling of each patient, we applied four inverse problem methods using Brainstorm toolbox solution. We implemented investigated inverse methods on averaged pure transitory events. Averaged pure transitory are obtained by realigning events compared to global field power (GFP). Then, we proceeded as in [5] to define active region as local peaks of source activation film. We explored all resulted local peaks as regions of interest ROI and nodes of connectivity networks graphs. Inversion was resulted as a single signal for each considered active region ROI.

Functional connectivity was estimated using cross-correlation coefficients as in [5]. We imposed lags in this range [-50, 50] ms, then we kept only the lag corresponding to a maximum correlation; the lag sign is used to define link directionality. Moreover, we applied a non-parametric method (Surrogate data) to threshold graphs. 1000 surrogate correlations realizations are generated and we retained only the maximum across pairs for each realization. Finally we picked the threshold value from resulting histogram corresponding to p =0.05. However, obtained ROI by MNE, dSPM, eLORETA and cMEM proved differences in amplitude and spatial extend and hence obtained functional connectivity too. An essential question arises at this level: which network connectivity is the most significant to assist neurologists in designation of EZ or during pre-surgical evaluation?

Simulation of brain connectivity could evaluate these results, but it remains non-sufficient, in epilepsy due to complexity of correlation and distribution between neurons. Remain; intracerebral network connectivity of pure epileptic transitory could be more decisive to validate epileptic MEG network connectivity. Since IEEG can offer an exclusive sequence of high spatiotemporal resolution and causal cortical information essential in defining EZ.

We measured cross-correlation between epileptic transitory sources (ROI as a node) for MEG connectivity. However, for IEEG connectivity graphs, we selected visually exact contact of pure epileptic transitory. Then, we measured cross-correlation (as in MEG) between these contacts as nodes of IEEG graphs. We obtained networks depicting 7 to 15 nodes (depending on studied subject), illustrating selected ROI (as potential source of pure epileptic transitory). Each node could be connected to one or more nodes within a link obtained from cross-correlation measure. Node degree presents number of connections of actual node toward the rest of nodes. Connection Strength illustrates the amplitude of connection between nodes (cross-correlation measures between active regions/nodes). Average Propagation delay depicts average amount of time required for excessive discharges to travel from a node to another one.

## 3. Results

### 3.1. Recovered Simulated Pure Transitory Events

In Figure 1, we depict one realization for SNR = 10 dB of simulated data. There is a mixture between transitory and ripples for different levels of overlap and time occurrence of epileptic transitory activities. We obtained 5 noisy channels; each one presents an overlap between transient and ripples (with frequency of 45 Hz, 55 Hz, 65 Hz, 75 Hz, and 85 Hz).

In Figure 2, we present transitory activity detection using local peaks.

In Figure 3, we illustrate recovered pure transitory among ripples of 85 Hz by projecting original signal on transitory basis obtained by our proposed advanced filtering technique.

In Figure 4, we depict robustness of recovering noncontaminated transitory activities among ripples of 45, 55, 65, 75, and 85 Hz and for three SNR values of -5, 10, and 20 dB.

GOF is computed between original simulated transitory and recovered pure transitory (noncontaminated by ripples). Increasing frequency and SNR values improved the performance of GOF. For low gamma, GOF is about 80%, which reaches 90% of resemblance for 85 Hz oscillations. For low SNR, GOF would not exceed 60% of reconstruction; however, for 20 dB of SNR, the GOF reach 93% of resemblance.

These results (effect of frequency range and SNR on the capacity of separation between transient and ripples activities) were in agreement with a previous work for other type of electrophysiological signals [8, 11, 24, 38].

### 3.2. Recovered and Detected Pure Transitory among MEG Signals

In Figure 5, we illustrate studied MEG signal recorded on 151 captors (we highlighted only 31 captors). MEG signal depicts three kinds of activity: oscillations (for different rhythms), transitory, and patterns made-up of a mixture between transitory and ripples (selected by an expert neurologist).

In Figure 6, we present transitory activity clustering results among MEG signals; two groups of transitory activities are eclectic. The first group is made of transitory events from epochs 1 to 14; and the second cluster includes transitory events from epochs 24 to 34. The first cluster has initiated its start by a discharge state; however, the second cluster has finished by a discharge.

In Figure 7, we delineate reconstructing pure epileptic transient activities by projecting real signal on our suited transitory basis. All transitory activities were successfully recovered without oscillatory events: noncontaminated interictal epileptiform discharges.

In Table 2, we gathered precision of automatic detection and reconstruction of pure transient activities among four channels (these MEG channels depict high occurrence of epileptic transitory events according to expert neurologist).

Precision of automatic detection and reconstruction of pure transient varies from 81% to 87%. These results are very promising, in defining efficiently epileptogenic zone EZ. In agreement with a null hypothesis, which supposes epileptic transient, within a specific generators or sources.

In Figure 8, we depict topography map of averaged transitory events in the peaks timing (channel 25 presented in Figures 7) before and after applying our routines of automatic detection and reconstruction. Averaged pure epileptic transitory shows dipolar topography that reflects an accurate cerebral source responsible of excessive discharges. However, topography map of averaged mixed transitory and ripples display much random and complex activities that turned the definition of responsible sources as a difficult and hard task to explain physiologically. Hence, our advanced technique improved the characterization of excessive discharges sources, since topography map of reconstructed-transitory activities illustrates a dipolar activity (no further activation). This result will lead to a better recognition and delineating of accurate EZ.

### 3.3. Results of MEG Source Localization

In Figure 9, we depict active region (local peaks of source activation film) of pure transitory activities using MNE, dSPM, eLORETA, and cMEM inverse problem methods.

eLORETA shows the highest number of active regions ROI (about 15 ROI for patient 2) and the most spatially extended ROI followed by MNE and dSPM (the order between MNE and dSPM depends of studied patient). The lowest active regions are obtained by cMEM. Moreover, cMEM results were totally in concordance with MEM performances studies [36, 37] that proved efficiency of MEM techniques in detecting deepest sources.

After computing network connectivity of pure MEG epileptic transitory and intracerebral EEG, we collect several information in order to confront MEG networks with IEEG ones. We detail common nodes as similar selected cortical region or ROI obtained by both MEG and IEEG. We determine the ratio of detected IEEG nodes conformed in MEG and vice versa. Finally, we checked if MEG nodes recognize the region of Seizure On set Zone (SOZ) (from clinical report).

In Table 3, we gathered concordant nodes, SOZ, and nodes ratio detected by one modality and checked by second modality of registration and vice versa and average propagation delay.

Number of nodes in common among MEG and IEEG network connectivity of pure transitory clearly varies from 0 to 4. These common nodes define also a part of seizure onset zone. eLORETA and cMEM provide with 100% of efficiency at least one node of SOZ, followed by MNE and dSPM, with only 60% of robustness in recognition of SOZ. These concordant sources are an effective way to match noninvasive modalities versus invasive-ones (IEEG versus MEG). Furthermore, entire inverse techniques provided in an average of 73.5% for nodes detected in depth and confirmed by MEG and vice versa about 77.15% of node detected from MEG and seen in IEEG. We computed concordant node mean of connection strength using mean of absolute cross-correlation values represented in Figure 10.

There is 100% resemblance of concordant MEG and IEEG node connection strength obtained by MNE for 2 patients, dSPM, eLORETA, and cMEM for 1 patient. These results would reach four patients, when we analyze only connection strength. Hence, dSPM and eLORETA promote the propagation power of interictal epileptiform discharges due to its high connection strength. MNE proved a better characterization of connection strength between MEG and IEEG concordant Sources of Interictal epileptiform discharges.

In Figure 11, we depict the median distance between common MEG and IEEG nodes per studied inverse techniques and per subjects.

In addition, eLORETA and cMEM offer the closet sources to SOZ, since these concordant nodes define at least one part of SOZ for entire studied patients. eLORETA provides the most accurate position of EZ.

## 4. Discussion and Conclusions

Our first assumption in illustrating EZ with high accuracy is to study and source localize pure hallmark (pure transitory). In fact, transitory events may be generated by specific sources [9]. Hence, we validated firstly an advanced preprocessing technique based on SVD to separate transitory from ripples. Our evaluation of capability of separation on simulated data was based on GOF, which reached 93% of resemblance for 85 Hz and 20 dB. For MEG signal, we used topography maps to assess capacity of recognition and automatic detection of transient using our advanced methods. Our results were in concordance with previous works [8, 11, 24, 38]. In the second time, we proposed to estimate robustness of four distributed inverse problem methods: MNE, eLORETA, dSPM and cMEM in characterization and recognition of unhealthy cortical tissue: regions of excessive discharges. Hence, we applied MEG source localization on pure transitory events for 5 patients. We computed network connectivity among MEG and confronted to IEEG. We determined MEG and IEEG concordant nodes; we computed connection strength and distance between MEG and IEEG concordant nodes, their cooperation in recognition of seizure onset zone, and the average delay propagation of excessive discharge to travel from a ROI to another. MNE has the closet connection strength of networks comparing to IEEG ones. dSPM and eLORETA promote propagation power of interictal epileptiform discharges. cMEM proved a high matching between MEG network connectivity and intracerebral networks based on the distance between sources, followed by eLORETA, dSPM, and MNE. The closet sources to IEEG electrodes are obtained by dSPM about 18 mm. Average delay propagation of MEG is ranging in [18, 25]ms and for IEEG is between 12 to 22 ms. The entire method results were consistent with patient lesion. However, the size of networks, connection strength, degree, widespread, distance between sources obtained from a noninvasive technique versus IEEG, and average delay propagation vary from one inverse problem to another and from one patient to another. It is also, to mention, that no inverse problem network was identical to the IEEG network. This could be justified by the fact that several regions were not explored in IEEG. Furthermore, patients are still not seizure free yet, even after surgery intervention, which could be a positive clue of detected MEG ROI, that reinforces the MEG role in planning IEEG electrodes. Our obtained results could be considered a prognosis tool for distributed inverse problem of source localization. Nevertheless, it remains quite difficult to delineate accurate cerebral generators involved in excessive discharges and build-up of a seizure from only scalp MEG signal. The possibility to combine several registration techniques with functional MRI scanning (fMRI) may ameliorate recognition of epileptogenic zones. In addition, combining inverse problem methods or even making extra assumption in inverse method principle [39] can also be more effective in assisting a neurologist during epilepsy diagnosis. Another fertile track is to incorporate several hallmarks to transient activities, like ripples and high-frequency oscillations (HFOs) [40]. Potential strategy may be applied through merging network connectivity of different: modalities, hallmarks, and inverse problem techniques using firstly simulated data generators [41] (for hallmark and cortical sources), then realistic databases to enhance the definition and recognition of EZ.

## Figures and Tables

**Figure 1:** One realization of simulated data, five channels, which reproduce an overlap between transient and ripples.

**Figure 2:** Detection of transitory activities: in blue simulated data: a mixture between transient and ripples, red circle is low and high thresholding results to detect local peaks.

**Figure 3:** Line one: channel 5 of simulated data depicting a mixture of 85 Hz ripples and transitory activities; line 2: reconstruction of pure epileptic transitory activities.

**Figure 4:** GOF of recovered pure transitory among five ripples (45 to 85 Hz), for three SNR values of -5 dB (start of bars), 10 dB (blue circle), and 20 dB (end of bars).

**Figure 5:** In MEG signal (patient 1), 31 captors are highlighted depicting intermingled transitory activities and ripples; circle in red shows different shape of transitory activities.

**Figure 6:** Classification of patient 1 MEG transitory on two groups. Line 1: energy map of selected transitory for group 1 and 2; line 2: transitory cluster shapes.

**Figure 7:** Line 1 shows channel 25: a mixture of activities and rhythms and line 2 presents pure recovered transitory activities.

**Figure 8:** (a) Topography map on the peak of average original transitory; (b) topography map on the peak of average pure detected and reconstructed transitory activity (patient 1). A dipolar configuration for second map reflects a cerebral source.

**Figure 9:** Source localization of averaged pure epileptic MEG transitory using 4 inverse problem methods (cMEM, dSPM, MNE, and eLORETA).

**Figure 10:** Mean of connection strength between MEG and IEEG concordant nodes. The blue box illustrates the mean of MEG connection strength, and the green box depicts the IEEG mean of MEG connection strength, for studied inverse problem methods and per subject. MEG connection strength is higher than IEEG one; eLORETA and dSPM provide the highest connection strength. The red line defines the median of connection strength that varies from one patient to another and through inverse techniques.

**Figure 11:** Median distance between concordant MEG and IEEG nodes per studied inverse techniques and per subjects. The boxes define the median distance between concordant MEG and IEEG nodes; closet sources are obtained in this order by cMEM, eLORETA then dSPM, and finally MNE methods.

**Table 1:** Patient's clinical background.

Patients	Gender	Age	Structural magnetic resonance imaging (brain anatomy and pathology)	Epilepsy surgery	Treatment at the time of MEG recording
1	Female	17	Right lateral occipitotemporal Focal cortical dysplasias	Right occipitotemporal cortectomy	Phenytoin+lamotrigine+gabapentin
2	Female	26	Normal	Left occipitotemporal cortectomy	Phenytoin+clobazam (20 mg/day)+carbamazepine+phenobarbital (50 mg/day)
3	Female	25	Left premotor Focal cortical dysplasias	Left premotor cortectomy	Phenytoin+carbamazepine+levetiracetam
4	Male	25	Right basal occipitotemporal Focal cortical dysplasias	Right anterior temporal lobectomy	Lamotrigine+pregabalin
5	Female	31	Right parietal ischemia	Right parietal cortectomy	Carbamazepine+levetiracetam+clonazepam (1.5 mg/day)

**Table 2:** Precision of automatic detection and reconstruction of pure epileptic transitory events.

Channels	TP	FP	P
MLC14	194	28	87%
MLC15	187	32	85%
MLC33	201	46	81%
MLC43	198	38	83%

**Table 3:** Nodes in common per patient and inverse problem methods.

Methods	Patient	Number of nodes in common	SOZ	% of MEG nodes confirmed by IEEG	% of IEEG nodes confirmed by MEEG	Average propagation delay in ms
MNE	1	2	Yes	74.6%	79.8%	22
	2	0	No			21
	3	2	Yes			20
	4	0	Yes			25
	5	1	No			22

eLORETA	1	2	Yes	78%	80.2%	20
	2	1	Yes			19
	3	3	Yes			23
	4	2	Yes			18
	5	4	Yes			21

dSPM	1	1	No	71.4%	75.4%	22
	2	2	No			25
	3	1	Yes			25
	4	2	Yes			23
	5	2	Yes			22

cMEM	1	1	Yes	70%	73.2%	25
	2	1	Yes			23
	3	1	Yes			23
	4	1	Yes			19
	5	1	Yes			21

## Data Availability

The data that support the findings of this study are available from the supervised author (Nawel Jmail), upon reasonable request. Local ethical committees allow the authors to share the data.
